# ECG Signal Classification Based on Fusion of Hybrid CNN and Wavelet Features by D-S Evidence Theory

**DOI:** 10.1155/2021/4222881

**Published:** 2021-09-07

**Authors:** Jixiang Zhang, Chengqin Wu, Chenzhao Ruan, Rongxia Zhang, Zengshun Zhao, Xiangqian Cheng

**Affiliations:** College of Electronic and Information Engineering, Shandong University of Science and Technology, Qingdao 266590, China

## Abstract

At present, cardiovascular disease is regarded as one of the dangerous diseases that threaten human life. The morbidity and lethality caused by cardiovascular disease are constantly increasing every year. In this paper, we propose a two-stream style operation to handle the electrocardiogram (ECG) classification: one for time-domain features and another for frequency-domain features. For the time-domain features, convolutional neural networks (CNN) are constructed for feature learning and classification of ECG signals. For the frequency-domain features, support vector regression (SVR) machines are designed to perform the regression prediction on each signal. Finally, the D-S evidence theory is adopted to perform the decision fusion strategy on the time-domain and frequency-domain classification results. We confirm a recognition performance of 99.64% from the experiment result for the D-S evidence theory recognition system upon the MIT-BIH arrhythmia database. The analysis of various methods of ECG classification shows that the model delivers superior performance promotion across all these scenarios.

## 1. Introduction

Cardiovascular disease is a disease with the highest incidence and mortality of human noncommunicable diseases [1]; they are threatening the lives of millions of people. Therefore, it is of great significance to diagnose ECG signals efficiently and accurately. The ECG signals can monitor the rhythm of the heart's activity, and it is useful to monitor heart diseases [2]; it contains a wealth of basic physiological signals of the heart, so it is often used to detect physical health disorders. At present, the processing methods of ECG signals are mostly manual analysis, which is very tedious and time-consuming. With the continuous progress of deep learning, the efficiency of ECG analysis and processing has been greatly improved.

There are various methods to automatically detect and classify abnormal ECG signals, such as wavelets analysis [3], deep belief network (DBN), and support vector machine (SVM) [4]. For the time-domain features, Mehrdad Javadi et al. [5] used the complementary features of Mixture of Experts (ME) and Negatively Correlated Learning (NCL) to classify ECG signals; they obtained a recognition rate of 96.02%. Rajpurkar et al. [6] constructed a CNN model, which diagnoses 14 types of arrhythmias, and it achieved a high accuracy rate. Li et al. [7] employed a 1-dimensional CNN, they introduced SMOTE algorithm to augmented data and achieved 98.12% accuracy. Alif et al. [8] have developed a 2D CNN for extracting shape-related features to detect arrhythmia. In their study, the classifier contains six convolutional layers, and the method shows an accuracy of 94.37%. Marinho et al. [9] introduced Structural Co-Occurrence Matrix (SCM) to extract features for the first time, and it was demonstrated to be promising for ECG classification.

Due to the limitations of the time-domain methods, these methods just analyse the ECG signal in time domain, and the results are not very well. For the frequency-domain features, Faziludeen et al. [10] used wavelets and SVM for classification, and they achieved 98% accuracy, but they only identified two types of abnormal ECG signals. Radovan et al. [11] utilized PQ intervals and QRS complexes to extract features and used genetic algorithm to select features and train SVM. They obtained a recognition rate of 84%. To reduce the segmentation step, Mondéjar-Guerra et al. [12] constructed multiple SVMs for the ECG signal classification, each SVM trained with a different feature. Compared with a single SVM model, their approach offered a satisfactory performance, and they achieved 94.5% accuracy. The highlights and drawbacks of these papers are shown in Table 1.

D-S evidence theory can fuse the prediction results of multiple classification models of the predicted target, and it is usually applied to the fusion of the decision layer to perform the final reasoning and decision-making process. Zhang Lizhi et al. [13] have implemented CNN and D-S evidence theory for the gearbox composite fault diagnosis, and they obtained an accuracy of 84.58%. Moreover, Geng Changxin [14] has advanced a diagnosis model of fused gearbox fault by using the D-S evidence theory, and this method showed 90% accuracy.

Due to the limitation of time-domain signal analysis, some researchers use frequency-domain characterization information to assist the signal analysis process. Compared with the time-domain method, frequency-domain signal processing has many advantages. However, it is not enough to complete the signal classification tasks by frequency-domain processing alone, so the time information is complemented for more accurate correspondence. In this paper, we propose a novel way to integrate the estimation in the frequency domain (such as the wavelet packet) and in the time domain. Furthermore, compared with the single classifier, multiple classifier systems (MCS) are more robust and the classification accuracy is higher [15]. Motivated by fusion of multiple classifier systems, we proposed to fuse the estimation of the CNN classifier and the SVR output of the wavelet packets.

In this paper, we proposed a new classification system using 1D CNN and SVR to learn the hybrid heartbeat features, and incorporate the outputs by D-S evidence theory, as shown in Figure 1. The CNN has the advantage in high-level feature mining due to its complex network structure. For time-domain features, this paper builds 1D CNN to classify the ECG signals. For frequency-domain features, wavelet packets and multiple SVR machines are designed for frequency-domain feature learning and classification. Both 1D CNN and SVR have performed relatively well on ECG signals. The innovation of this paper is that D-S evidence theory is used to fuse the recognition results of 1D CNN and SVR, because the results come from different domains, and this method is beneficial to improve the accuracy. Compared with a single classifier, this method has a higher classification performance. In the end, we compare our method with previous work. The results show that the proposed method has better accuracy. The main contributions of the proposed method are as follows:

1. This paper proposed a novel multiclassifier ECG signal recognition framework; specifically, we utilize 1D CNN to extract time-domain features, and frequency-domain features are extracted by wavelet packet and classified by SVR. Then, we introduce the D-S evidence theory to fuse the recognition results of 1-D CNN and SVR, which obtains a better classification performance.
2. The introduction of D-S evidence theory can make up the singleness and incompleteness of feature extraction in a single domain.
3. Since the classification results of the classifier are derived from the time-domain and frequency-domain, the method in this paper achieves better performance than other methods in MIT-BIH dataset.

The remainder of this article is organized as follows. Methods are presented in Section 2, followed by the experimental design and classification models in Section 3. Experimental results and discussion of the proposed model are given in Section 4. Finally, this paper gives the conclusion and the future directions.

## 2. Materials and Methods

### 2.1. Dataset

In this paper, we used MIT-BIH Arrhythmia Database for experiment and analysis [16]. This database contains 48 different patient records obtained from 47 subjects and extracted from two leads (lead II (MLII) and lead VI). The lead II was used as the default as the QRS is more prominent. The label of ECG signals was annotated by multiple cardiologists independently; it can reduce the error in the diagnoses. In this paper, five ECG signal categories are considered; each segment has one beat type, which consists of 250 samples. The created fragments contain 99 samples before the R peak and 150 samples following the R peak.  Table 2 shows the details of the ECG signals in this study; the typical ECG segments of A, *L*, R, V, and N signals are shown in Figure 2.

### 2.2. ECG Signal Preprocessing

Initially, ECG signals that obtained from MIT-BIH dataset contain low frequency and high frequency, such as machine interference [17] and muscle movement. For the low-frequency noise, we use the mean filtering and median filtering algorithm, and the effect of median filtering is generally better than mean filtering, so this paper used the median filtering algorithm to get rid of low-frequency noise, and the median filter window size was set to 50 and 150 steps [18]. For the high-frequency noise, we studied an approach to eliminate the power frequency interference from ECG signals based on wavelet transform. The method of the soft threshold is adopted to analyse the wavelet coefficient. It can effectively remove the high-frequency noise and retain the original features of ECG signals.  Figure 3 shows the original and reconstructed ECG signal.

### 2.3. R-Wave Detection and Segmentation

Having removed the noise, the ECG signals need to be segmented by waveform detection. In this paper, we utilize the QRS waves to segment ECG signals. Since the QRS complex is a dominant feature and a crucial part of ECG signals, we use the difference threshold algorithm [19] to detect QRS waves. This algorithm contains the operation of difference, square, and moving window integration, which correspond to formulas (1)–(3) [19], respectively. Finally, the R-wave was extracted through the legal position of the dual threshold method (formulas (4) and (5)) [19].

(1) $$\begin{array}{c} y\left(n\right)=\frac{1}{8}\left[2x\left(n+1\right)-x\left(n-1\right)+x\left(n+2\right)-x\left(n-2\right)\right], \end{array}$$

(2) $$\begin{array}{c} y\left(n\right)={\left[x\left(n\right)\right]}^{2}, \end{array}$$

(3) $$\begin{array}{c} y\left(n\right)=\frac{1}{N}\left[x\left(n-\left(N-1\right)\right)+x\left(n-\left(N-2\right)\right)+x\left(n-\left(N-3\right)\right)...+x\left(n\right)\right], \end{array}$$

where *x*(*n*) is the input ECG signal, *y*(*n*) is the output signal, *n* is the point of the difference operation, and *N* is the width of the moving window.

(4) $$\begin{array}{c} \text{TH}1=\text{NPKI}+0.25\left(\text{SPKI}-\text{NPKI}\right), \end{array}$$

(5) $$\begin{array}{c} \text{TH}2=\text{0.}5\left(\text{TH}1\right). \end{array}$$

where TH2 and TH1 are high threshold value and low threshold value, respectively. SPKI is the value of the QRS peak, and NPKI is the first value of the noise peak.

Then, the locations of the QRS wave were marked in the original signal time domain. Based on the MIT-BIH sampling rate of 360 Hz, the R-wave was used as the benchmark. The final decision was made to take 100 points to the left and 150 points to the right, respectively; that is, the 250 points contain a complete beat sample.  Figure 4 shows an individual heartbeat waveform of the ECG signal sample.

### 2.4. Feature Extraction

In the time domain, the 1D CNN model is applied to automatically extract features from preprocessed ECG signals. After the signals are detected and segmented into individual waveforms, we can obtain plenty of complete time-domain features, including P wave, QRS wave, and T wave. The arrhythmia types of each ECG signal in the MIT-BIH database have been labeled by medical experts. The 10-fold cross-validation is employed in this study, and the average result of all the 10 folds was calculated as the final performance of the system. As shown in Table 2, we choose five types of heart arrhythmia: N, R, L, V, and A; then we randomly select 2000 samples from each type as the sample set: 90% of them as the training sample set, and 10% samples as the test set. Then, we use a 1D CNN for classification; it contains four convolution layers, four max-pooling layers, and a fully connected layer.

The wavelet packet analysis technique is utilized in the frequency domain, and it can be well applied to ECG signal processing in time-frequency analysis; it provides a more detailed method to signal analysis. As is shown in Figure 5, the wavelet packet can decompose the high-frequency part finer than the wavelet transformation. Moreover, according to the characteristics of the ECG signals, it can select the corresponding frequency band adaptively and make it match with the signal spectrum, so as to improve the time-frequency resolution. In this paper, we utilize Daubechies 6 (db6) [20] as the wavelet basis to decompose the signals in five scales and obtain 32 wavelet packet coefficients, including the high-frequency components of ECG signals. Then, we extract the variance, mean, and maximum value of the 32 coefficients as the ECG signals transformation domain features. SVR is used to train the classification features of five arrhythmia types. The sample set is the same as that of CNN.

## 3. Construction and Fusion of the Classification Model

In this section, we proposed a novel framework to automatically recognize five classes of arrhythmias. This hybrid system combines 1D CNN with wavelets features to meet this requirement. The classification results of these two models are fused by D-S evidence theory.

### 3.1. Classification Model Based on 1D CNN

CNN is a popular artificial neural network [21], because of its high learning efficiency; it has been widely used in the field of image recognition and achieved great success [22]. In the 1990s, Le Cun et al. [23] designed and trained the most classic CNN model, Lenet-5. The CNN model is composed of the input layer, convolutional layer, pooling layer, full connection layer, and output layer [24], the convolutional layer and pooling layer are arranged alternately, and this special structure can simplify the network parameters and makes CNN have translational and rotational invariance [25].

#### 3.1.1. Convolution Layer

The convolutional layer consists of multiple feature maps, each feature map is composed of multiple neurons, and each neuron is connected to the local area of the previous feature map through the convolution kernel. The function of the convolution layer is to learn the characteristic representation of the input data, enhance the information of the original data, and suppress the noise. The convolutional layer reflects the advantages of local connection and weight sharing [26]. In convolution, the network will learn features automatically without manually selecting features [26]. The convolution layer is calculated by the following formula [27]:

(6) $$\begin{array}{c} X_{\text{j}}^{l}=f\left(\sum_{i\in M_{j}}X_{i}^{l-1}*K_{ij}^{l}+b_{j}^{l}\right), \end{array}$$

where *X*_j_^*l*^ represents the *j*-th characteristic graph of the layer *l*, *K*_*ij*_^*l*^ is the convolution kernel function, *f*() is the activation function, *b*_*j*_^*l*^ is the bias parameter, and *M*_*j*_ represents the set of selected input feature graphs.

#### 3.1.2. Max-Pooling Layer

By reducing the resolution of the feature surface and the number of parameters, the max-pooling layer can obtain spatially invariant features. The max-pooling layer plays an auxiliary role in feature extraction. In this paper, we utilize the max-pooling operation to calculate the max value of a nearby set of inputs. It is defined as

(7) $$\begin{array}{c} X_{j}^{l}=f\left(\beta_{j}^{l}\max\left(X_{j}^{l-1}\right)+b_{j}^{l}\right). \end{array}$$

Here, max() is the max sampling function, and the size of the sampling window is *n* × *n*. Then, the output feature map is reduced by *n* times. Each output feature graph has its multiplicative bias parameters *β* and additive bias parameters *b*.

Finally, after alternating the convolution layer and pooling layer, SoftMax regression is adopted to return the probability of input data belonging to a certain category.

In the CNN classifier, the convolutional layer and the max-pooling layer are alternately connected to generate a deep neural network, which can efficiently extract the basic features of ECG signals. The ECG signals belong to one-dimensional discrete data, so it is necessary to build 1D CNN.  Table 3 shows the layer details and the parameters of 1D CNN.

### 3.2. Classification Model Based on SVR

SVM technique is a classical machine learning method proposed by Vapnik and co-workers [28]. This technology has been further modified in various fields. As a kind of model for SVM to deal with fitting problems, support vector regression (SVR) can predict the test data by establishing the nonlinear relationship between the support vector and the predicted vector in the training data; SVR solves the problem of nonlinear fitting well by introducing kernel function to replace the calculation of high-dimensional space and regression. The regression function in the feature space is expressed as [29]

(8) $$\begin{array}{c} f\left(x\right)=w^{T}\phi \left(x\right)+b, \end{array}$$

where *ϕ*(*x*) is the feature space, *w* is the weight parameter, and *b* is the bias parameter. According to the structural risk minimization principle, and introducing relaxation variables, *w* and *b* can be minimized to obtain the following objective function [29]:

(9) $$\begin{array}{c} R\left(w,\xi_{i},\xi_{i}^{*}\right)=\frac{1}{2}{\left\|w\right\|}^{2}+C\sum_{i=1}^{l}\left(\xi_{i}+\xi_{i}^{*}\right), \end{array}$$

which is subject to the constraints

(10) $$\begin{array}{c} y_{i}-w\phi \left(x_{i}\right)-b\leq \varepsilon +\xi_{i},\\ w\phi \left(x_{i}\right)+b-y_{i}\leq \varepsilon +\xi_{i}^{*},\\ \xi_{i},\;\xi_{i}^{*}\geq 0,\;i=1,2,\ldots ,l. \end{array}$$

where *C* and *ε* are the prescribed parameters, 1/2‖*w*‖^2^ measures the flatness of the functions, and *C* represents the trade-off between the flatness and empirical risk.

In this paper, the ECG signal is broken down into five scale wavelet packets, and we obtained 32 wavelet packet coefficients, which make up the sample space. Besides, we constructed five subclassifiers for ECG signals classification. Each classifier is trained to classify one ECG signal type as a positive sample and the rest as negative samples. After the training step, each classifier can output the probability of the classification result of the test sample.

In this paper, we propose SVR for classification. Kernel functions of SVR include polynomial kernel function, linear kernel function, multilayer perceptron, and radial basis kernel function. The extracted transform domain features, namely, 96 wavelet statistical features, are normalized and composed into a sample set. We utilize the radial basis kernel function for classification. This kernel function has two parameters: the kernel parameter *g* and the penalty parameter *c*. The optimal parameters of *g* and *c* are obtained by cross-validation, and the results are *g*  = 3.2 and *c* = 2.9.

### 3.3. Incorporation by D-S Evidence Theory

#### 3.3.1. Principle of Evidence Theory

D-S evidence theory is an uncertainty inference theory proposed by Dempster in 1967 and further developed by his student Shafer. It can deal with the uncertainty of results effectively and the fusion of multiple classifier data results [30]. The basic principle of D-S evidence theory is to define the frame Ω, which is usually a finite set; it is a set of incompatible basic propositions or assumptions about the problem. In general, all subsets of Ω are represented as power 2^Ω^, and the basic probability distribution is defined as follows [31].

**Definition 1 .**

(see [31], basic probability distribution). If *m*(*A*) satisfies the mapping from 2^Ω^ to [0,1] in the frame of discernment, and *A* stands for any subset of Ω, then it satisfies

(11) $$\begin{array}{c} \left\{\begin{array}{c} m\left(\Phi \right)=0,\\ \sum_{A\in \Omega }m\left(A\right)=1. \end{array}\right) \end{array}$$

Then, *m* is the basic probability assignment function (BPAF) on the Ω.

**Definition 2 .**

(see [31]). *m*(*A*) is the trust function, and it is usually utilized to define the lower bound of probability. The upper limit of probability can be determined by the likelihood function. The belief function (Bel) and plausibility function (Pls) are shown in the following formula:

(12) $$\begin{array}{c} \text{Bel}\left(\text{A}\right)=\underset{B\subseteq A}{\sum }m\left(B\right),\\ \text{Pls}\left(A\right)=1-\text{Bel}\left(\bar{A}\right). \end{array}$$

Bel(A) and Pls(A) are calculated to form the trust interval [Bel(*A*) , Pls(*A*)] to indicate the degree of certainty of a hypothesis.

#### 3.3.2. Evidence Theory Fusion of CNN and SVR Classifier Results

In this paper, we propose a two-stream style operation to handle the electrocardiogram (ECG) classification: one for time-domain features (the features are obtained and classified by CNN) and the other stream for frequency-domain features (the features are obtained by wavelet packets and classified by SVR). The fusion of CNN and SVR classifier belongs to the fusion of two evidences. The formula of the composition rules [31] is as follows:

(13) $$\begin{array}{c} m\left(A\right)=\frac{\sum_{A_{i}\cap B_{j}=A}m_{1}\left(A_{i}\right)m_{2}\left(B_{j}\right)}{1-\sum_{A_{i}\cap B_{j}=\phi }m_{1}\left(A_{i}\right)m_{2}\left(B_{j}\right)}, \end{array}$$

where *m*_1_ and *m*_2_ are the probability distribution functions of the predicted results of CNN and SVR for the same test sample and *A*_1_ ~ *A*_5_ and *B*_1_ ~ *B*_5_ are the corresponding focal elements, respectively.

## 4. Results and Discussion

### 4.1. Experimental Setting

The experimental software is MATLAB R2018a, and the hardware environment is Intel i7-10875H processor, 16 GB memory, Windows 10 operating system. The model is trained for 600 epochs each time, and the batch size is set as 64. We used the adaptive moment estimation (Adam) to update the CNN weights, and the initial learning rate was 0.01.

In this paper, a 10-fold cross-validation is employed, and the average result of all the 10 folds was calculated as the final performance. We use the positive predictivity (PPV), sensitivity (SEN), specificity (SPE), and accuracy (Acc) to evaluate the effectiveness of the model. Moreover, *F*1-score is used to evaluate the model; the formulas are as follows:

(14) $$\begin{array}{c} \mathrm{PPV}=\frac{\sum_{i}^{N}\text{TP}/\text{TP}+\text{FP}}{N}\times 100\%,\\ \mathrm{SE}=\frac{\sum_{i}^{N}\text{TP}/\text{TP}+\text{FN}}{N}\times 100\%,\\ \mathrm{SP}=\frac{\sum_{i}^{N}\text{TN}/\text{TN}+\text{FP}}{N}\times 100\%,\\ \mathrm{Acc}=\frac{\sum_{i}^{N}\text{TP}+\text{TN}/\text{TP}+\text{FP}+\text{TN}+\text{FN}}{N}\times 100\%,\\ F\mathrm{1-score}=\frac{\sum_{i}^{N}2\text{TP}/2\text{TP}+\text{FP}+\text{FP}}{N}\times 100\%. \end{array}$$

where N represents the number of sets applied in the 10-fold and TP, TN, FP, and FN are true positives, true negatives, false positives, and false negatives, respectively.

### 4.2. Experimental Results and Analysis

The performance of different classifiers is mainly compared in this section. We use Acc as the evaluation indicator to compare the performance differences of 1D CNN, SVM, and the fusion of them by D-S evidence theory (D-S model). The classification results are presented in Tables 4–6.

We utilize 1D CNN and SVR to classify five types of ECG signals. The prediction results are shown in Tables 4 and 5.

The achieved results reported in Table 4 show that 1D CNN model successfully classifies the ECG signal. The *F*1-scores of *N* and *L* are relatively high, reaching 99.34% and 99.65%. The *F*1-score of *A* is low, only 97.43%, and the overall Acc of the model is 99.50%.  Table 5 shows that the *F*1-scores of R and *L* are higher than others. The *F*1-score of *A* is relatively low, only 90.12%, and the overall Acc is 96.46%.

The results of 1D CNN and SVR model are fused by D-S evidence theory.  Figure 6 shows the final confusion matrix of this classification system.

Table 6 shows that the *F*1-scores of *R* and *L* are relatively high, reaching 99.98% and 99.76%. The A is low, only 98.20%, and the overall accuracy rate of the model is 99.64%; it is generally increased nearly 0.14%.  Table 7 lists the 16 metrics of classification results, including PPV, SE, and SP of each beat and the average Acc. The D-S model has the best comprehensive classification ability: yielding 11 highest scores on 16 metrics. It achieves the best average *F*1-score and Acc of 99.3% and 99.6%. From Table 6 and Table 7, it can be deduced that the D-S evidence theory improved the performance of classification.

As can be seen from Figure 7, the recognition rate of the evidence-based fusion method is better than that of the 1D CNN and SVR classifiers; it has a high and stable recognition accuracy.

In summary, the classification performance of the method is superior to those listed in Table 8 in the task of ECG signal classification. In our study (marked in bold, Table 8), the classification proposed in this paper is different from other studies. This method utilizes D-S evidence theory to fuse the classification results of 1D CNN and SVR to obtain the final classification results. The experiment proves that, by introducing the D-S evidence theory, the multiclassifier system can be more robust and improve the classification accuracy effectively.

The main advantages of our proposed system are summarized as follows:

1. We utilize 1D CNN and wavelet packet to extract time-domain and frequency-domain features, respectively. Then, we introduce the D-S evidence theory to fuse the recognition results, which obtain better classification performance.
2. This method uses the 10-fold cross-validation approach. Hence, the results reported are robust.
3. This method makes up the singleness and incompleteness of feature extraction in a single domain.

The drawbacks of our proposed model are as follows:

1. Classification of ECG signals needs to be improved, such as AAMI classification.
2. This method cannot deal with negative peaks effectively.

## 5. Conclusions

This paper proposed an innovative method for ECG classification, which combines 1D CNN and SVR. The proposed method has good generalizability in nature, and this method can effectively deal with the classification problem in biomedical applications. 1D CNN classifier is constructed in the time domain for feature learning. The SVR classifier is constructed in the frequency domain for five scale wavelet packet decomposition of ECG signals; then we obtained 32 arrays of wavelet packet systems to construct the sample space. Finally, we used D-S evidence theory to fuse the predicted results of 1D CNN and SVR classifier, and the recognition accuracy is further improved. One of the most significant contributions of this study is that we propose D-S evidence fusion to classify ECG signals. To our knowledge, this is the first effort to use D-S evidence fusion for ECG signal detection. The classification accuracy of the proposed model reached 99.64%. In the future, we intend to improve the method of preprocessing ECG signals to solve the problem of negative peaks. Moreover, we will try to recognize more types of ECG signals in different datasets.

## Figures and Tables

**Figure 1:** The framework of the proposed classification model.

**Figure 2:** Waveforms of five arrhythmia types: (a) A, (b) L, (c) R, (d) V, and (e) N.

**Figure 3:** Renderings of low-frequency and high-frequency noise suppression.

**Figure 4:** An individual heart beat waveform of the ECG signal sample.

**Figure 5:** The structure diagram of wavelet packet decomposition [20].

**Figure 6:** Confusion matrix of the classified ECG signals.

**Figure 7:** Comparison of accuracy of three models.

**Table 1:** The main highlights and drawbacks of the methods mentioned.

Author	Approach	Database	ECG beats	Advantages	Disadvantages
Balasundaram [3]	Wavelet analysis	MITDB	Rhythmic ventricular tachycardia WA (VT) Organized ventricular fibrillation (OVF) Disorganized ventricular fibrillation (DVF)	This method performs well in the overlap zone between VT and VF.	The limitation is that it cannot be used as a risk-stratifier, because this method cannot determine the probability of future VF episodes.

Sayantan [4]	Gaussian-Bernoulli deep belief network and active learning	SVDB MITDB	AAMI	By using the expert interaction, this method is robust and it can overcome the variance in data distribution in interpatient scenarios.	This method handles intraclass variations poorly.

Javadi [5]	ME and NCL	MITDB	Normal (N) Premature ventricular contraction (PVC) Others	Combined with NCL and ME, it can enable the training algorithm of ME to establish a balance in bias-variance-covariance trade-offs, and it improves the accuracy and generalization of the model.	This work does not provide further insights of the classification boundaries.

Rajpurkar [6]	CNN	MITDB	Atrial fibrillation (AFIB) Atrial flutter (AFL) Complete heart block (CHB) Ectopic atrial rhythm (EAR) (14 rhythm types), etc.	This method uses a very deep CNN; the model can achieve a high accuracy rate under a big dataset. It can be used for a single-lead wearable monitor.	If two ECG signals are similar, the model sometimes makes mistakes, such as Wenckebach and AVB_Type2, Supraventricular Tachycardia (SVT), and atrial flutter (AFL).

Li [7]	CNN	MITDB	AAMI	This method uses the SMOTE algorithm to balance the classes in dataset.	It only extracted the time-domain features.

Alif [8]	2D CNN	MITDB	AAMI EC57	This method utilizes CNN to extract features automatically.	It only extracted the time-domain features.

Marinho [9]	Feature extraction: Fourier, goertzel, higher order statistics (HOS), and SCM. Classifier: support vector machine, multilayer perceptron, bayesian, and optimum-path forest	MITDB	ANSI/AAMI AAMI2	This is the first time that SCM has been applied to feature extraction. This paper combines different feature extraction methods, the accuracy is improved, and the classification rate is relatively high.	It is dependent on QRS's window lengths.

Faziludeen [10]	Wavelets and SVM	MITDB	Normal (N) Premature ventricular contraction (PVC) Left bundle branch block (LBB)	This work uses one against one (OAO) SVM to classify ECG signals.	This method requires designing features manually, and the classification of ECG signals is less.

Radovan [11]	SVM	PhysioNet/CinC	Normal (N) Atrial fibrillation (A) Other rhythm (O) Noisy records (P)	Combined with SVM and simple threshold-based rules, it can improve performance.	This method requires designing complex features manually.

Mondéjar-Guerra [12]	Multiple SVMs	MITDB	Normal (N) Supraventricular ectopic beat (SVEB) Ventricular ectopic beat (VEB) Fusion (F)	This work trains and integrates specific SVM models for each type of feature; it offers a satisfactory performance.	Data fusion is relatively simple.

**Table 2:** The type of arrhythmia used in this paper.

Classes (instances)	Size of segments
Atrial premature beat (A)	2545
Left bundle branch block (L)	8068
Right bundle branch block (R)	7254
Premature ventricular contraction (V)	7026
Normal (N)	74955
Total	99848

**Table 3:** The architecture of 1-D CNN.

Layers	Type	Activation function	Number of neurons (output layer)	Filter size	Number of filters	Stride
1	Input		250 × 1			
2	Convolution	ReLU	246 × 4	5 × 1	4	1
3	Max-pooling		123 × 4	2 × 1	4	2
4	Convolution	ReLU	120 × 4	4 × 1	4	1
5	Max-pooling		60 × 4	2 × 1	4	2
6	Convolution	ReLU	56 × 4	5 × 1	4	1
7	Max-pooling		28 × 4	2 × 1	4	2
8	Convolution	ReLU	24 × 8	5 × 1	8	1
9	Max-pooling		12 × 8	2 × 1	8	2
10	Fully connected	ReLU	10			
11	Output	SoftMax	5			

**Table 4:** Results of classification based on 1D CNN.

Type	*F*1-score	Acc (%)	PPV (%)	SE (%)	SP (%)
N	99.34	99.74	99.14	99.54	99.79
V	98.31	99.32	98.48	98.13	99.61
R	99.08	99.59	98.82	99.15	99.70
L	99.65	99.86	99.49	99.81	99.88
A	97.43	98.97	97.79	97.08	99.45

**Table 5:** Results of classification based on SVR.

Type	*F*1-score	Acc (%)	PPV (%)	SE (%)	SP (%)
N	90.04	95.86	86.23	94.24	96.27
V	95.49	98.27	97.92	93.21	99.51
R	97.18	98.88	97.38	97.00	99.35
L	97.35	98.92	96.27	98.46	99.04
A	90.12	96.17	93.20	87.27	98.40

**Table 6:** Results of classification based on the incorporation of outputs by D-S evidence theory.

Type	*F*1-score	Acc (%)	PPV (%)	SE (%)	SP (%)
N	99.49	99.80	99.49	99.49	99.88
V	99.04	99.60	99.52	98.56	99.87
R	99.98	99.60	99.49	98.48	99.88
L	99.76	99.90	99.51	100	99.87
A	98.20	99.30	97.45	98.96	99.38

**Table 7:** Results of all classifiers on the ECG test dataset.

Classifier	Acc	N			V			R				L				A		
		PPV	SE	SP	PPV	SE	SP	PPV	SE	SP	PPV		SE	SP	PPV		SE	SP
1D CNN	99.5	99.1	99.5	99.7	98.5	98.1	99.6	98.8	99.2	99.7	99.4		99.8	99.9	97.8		97.1	99.5
SVR	96.5	86.2	94.2	96.3	97.9	93.2	99.5	97.4	97.0	99.4	96.3		98.5	99.0	93.2		87.3	98.4
D-S	99.6	99.5	99.4	99.8	99.5	98.6	99.9	99.5	98.5	99.9	99.5		100	99.8	97.5		99.0	99.4

**Table 8:** Comparison of different classification approaches.

Author	ECG beats	Approach	Database	Performance (%)
Mehrdad Javadi et al. [5]	Normal (N) Premature ventricular contraction (PVC) Others	Mixture of experts (ME) and negatively correlated learning (NCL)	MIT-BIH	SPn = 98.01 SEpvc = 92.27 SEother = 93.72 Acc = 96.02

Mondéjar-Guerra V [12]	Normal (N) Supraventricular ectopic beat (SVEB) Ventricular ectopic beat (VEB) Fusion (F)	SVMs	MIT-BIH	SEN = 95.9 PPVN = 98.2 SESVEB = 78.1 PPVSVEB = 49.7 SEVEB = 94.7 PPVVEB = 93.9 SEF = 12.4 PPVF = 23.6 Acc = 94.5

Shi hangrui [32]	Left bundle branch block (LBBB) Right bundle branch block (RBBB) Atrial premature beat (APB) Premature ventricular contraction (PVC)	Learning vector quantization (LVQ)	MIT-BIH	AccAPB = 84.2 AccPVC = 92.6 AccLBBB = 77.8 AccRBBB = 81.4 Acc = 84

Wang Run [33]	N LBBB RBBB PVC	Radial basis function (RBF)	MIT-BIH	AccN = 89.7 AccLBBB = 97.1 AccRBBB = 96.7 AccPVC = 93

Yıldırım et al. [34]	13 classes 15 classes 17 classes	CNN	MIT-BIH	SE13 = 93.52 SP13 = 99.61 PPV13 = 92.52 Acc13 = 95.2 SE15 = 88.57 SP15 = 99.39 PPV15 = 90.48 Acc15 = 92.51 SE17 = 83.91 SP17 = 99.41 PPV17 = 89.52 Acc17 = 91.33

Li et al. [35]	AAMI	RF	MIT-BIH	SEN = 94.67 PPVN = 99.73 SES = 20.00 PPVS = 0.16 SEV = 94.20 PPVV = 89.78 SEF = 50.00 PPVF = 0.52 SEQ = 0.00 PPVQ = 0.00 Acc = 94.61

Amrita Rana et al. [36]	N LBBB RBBB APB PVC	LSTM	MIT-BIH	Acc = 95.00

Anika alim et al. [37]	N abnormal	SVM and ANN	MIT-BIH	AccSVM = 87 AccANN = 94

Sherin M. Mathews et al. [38]	SVEB VEB	Restricted Boltzmann machine (RBM) and deep belief networks (DBN)	MIT-BIH	AccSVEB = 93.63 AccVEB = 95.87

Ours	N V R L A	CNN and SVR by D-S evidence theory	MIT-BIH	SEN = 99.49 SPN = 99.88 PPVN = 99.49 AccN = 99.49 SEV = 98.56 SPV = 99.87 PPVV = 99.52 AccV = 99.04 SER = 98.48 SPR = 99.88 PPVR = 99.49 AccR = 99.98 SEL = 100 SPL = 99.87 PPVL = 99.51 AccL = 99.76 SEA = 98.96 SPA = 99.38; PPVA = 97.45 AccA = 98.20 Acc = 99.64

## Data Availability

The MIT-BIH Arrhythmia Database used to support the findings of this study is publicly available and can be downloaded at https://physionet.org/content/mitdb/1.0.0/.
